This article has been retracted.

# Effects of the medicinal plant, *Tamarindus indica,* as a potential supplement, on growth, nutrient digestibility, body composition and hematological indices of *Cyprinus carpio* fingerlings

**DOI:** 10.1016/j.heliyon.2024.e33901

**Published:** 2024-06-29

**Authors:** Mahnoor Saleem, Syed Makhdoom Hussain, Shafaqat Ali, Muhammad Rizwan, Khalid A. Al-Ghanim, Jean Wan Hong Yong

**Affiliations:** a Fish Nutrition Lab, Department of Zoology, Government College University Faisalabad, Punjab, 38000, Pakistan; b Department of Environmental Sciences, Government College University, Faisalabad, Punjab, 38000, Pakistan; c Department of Biological Sciences and Technology, China Medical University, Taichung, 40402, Taiwan; d Department of Zoology, College of Science, King Saud University, Riyadh, 11451, Saudi Arabia; e Department of Biosystems and Technology, Swedish University of Agricultural Sciences, 23456, Alnarp, Sweden

**Keywords:** Fish growth, Carcass, Hematology, Digestibility, Plant Extract

## Abstract

*Tamarindus indica*, a beneficial herb, has many health benefits but there is limited research on its use in fish nutrition industry. The current study investigated the effects of incorporating extracts of *T. indica* into the canola meal-based diets of *Cyprinus carpio* (common carp); following which, the growth, digestibility, carcass and hematological markers were assessed. A total of six diets were formulated with varying concentrations of *T. indica* extracts (TIE) viz, 0 %, 0.5 %, 1 %, 1.5 %, 2 % and 2.5 %. The fish (N = 270, 15 fish/tank with triplicates) in each tank were fed experimental diets for 70 days. The study demonstrated that TIE supplementation significantly improved the growth of common carp when compared to 0 % TIE level (control). The best results were observed at 1 % TIE level for the specific growth rate (1.68 ± 0.03 %), weight gain (15.00 ± 0.57 g), and feed conversion ratio (1.36 ± 0.05). Conversely, the 2.5 % TIE level gave the least improvement in terms of growth performance. Specifically for nutrient digestibility, the maximum values of crude protein (CP, 67.60 ± 0.83 %), crude fat (CF, 67.49 ± 0.45 %) and gross energy (GE, 70.90 ± 0.56 %) were recorded at 1 % TIE level. In addition, the best results of body composition (protein: 63.92 ± 0.06 %, ash: 18.60 ± 0.03 %, fat: 7.12 ± 0.02 % and moisture: 10.36 ± 0.04 %) and hematological indices, were measured in carps fed with 1 % supplementation level. In conclusion, the overall health of *C. carpio* fingerlings was improved with TIE supplementation in the diet containing 1 % TIE.

## 1 Introduction

Fishes have a significant role in human society in terms of providing abundant sources of protein nutrition [1,2]. It has a high protein level and low-fat content, which makes it a healthy choice for human meals. Furthermore, it is an excellent source of omega 3 fatty acids. Fish farming is currently the fastest-growing sector of the food industry [[3], [21], [61]]. However, large-scale aquaculture is usually susceptible to disease outbreaks, resulting in reduced fish growth and productivity [[4], [5], [6], [7]].

In order to control disease outbreaks, antibiotics were employed to enhance fish's resistance to diseases, reduce inflammation and promote their growth and appetite [6]. However, the use of antibiotics raises concerns about food safety and human health as residual antibiotics persist in fish body [7]. Moreover, one significant negative effect of the extensive usage of antibiotics is the development of antimicrobial resistance [8].

Using natural prophylactic supplements in place of chemotherapy is seen to be an effective measure to strengthen fish immunity and also creating a healthy environment [[9], [61]]. Various botanicals and including Chinese herbal medicines may serve as a successful substitute for antibiotics due to abundance of bioactive components, including flavonoids, polysaccharides, saponins, polyphenols, essential oils, terpenoids and alkaloids [[10], [11], [62], [64], [65]]. These substances have been utilized extensively in improving growth, organ and tissue function, nutrient metabolism, controlling bacterial and viral infections [12].

One of the beneficial herbal supplement, tamarind tree or *Tamarindus indica* L, belongs to the Leguminosae (Fabaceae) family. It is a monotypic genus tree that originated in tropical Africa, but now, it is widely cultivated everywhere in the sub-tropics of the world [13]. Tamarind leaves, being edible, are used in making soups, salads and curries. Leaves are of about 5 cm, brightly green colored and arranged pinnately [14]. The chemical composition of the *T. indica* leaves includes, vitamins, proteins, lipids, and fibres [15]. Numerous phytochemicals have also been identified in this species, including flavonoids, benzyl benzoate, limonene, lupeol, luteolin, orientin, tartaric acid, palmitic acid, tamarindienal, cinnamaldehyde and terpenoids. Furthermore, these compounds are linked to the hepatoprotective, antihelmintic, antibacterial, wound-healing, antioxidant, antifungal and digestive effects of tamarind leaves [16]. Although *T. indica* leaves contain high levels of phytochemicals, there is little scientific information regarding their uses in the production of animal feed, especially for fishes [17]. According to some research efforts [17,18], feeding 1 % *T. indica* extract (TIE) and tamarind pulp extract to *Oreochromis niloticus* resulted in improved growth, physiology and digestion, respectively.

Common carp (*Cyprinus carpio*) is economically important fish for global aquaculture industry and has a broad distribution in natural freshwater environment [19]. It is a member of family Cyprinidae. This family, being on top of aquaculture production, accounts for approximately 18 metric tons of aquaculture production; It is also the largest freshwater fish family in the world [20]. Almost 4,189,500 metric tons of this species were produced commercially in 2018, making up 7.7 % of the global aquaculture production of finfish [21]. This fish species is considered to be popular farmed species and serving as a significant source of food [22]. Additionally, it is one of the most prominent species for aquaculture, contributing to ca 40 % of the world's farmed fish production. *C. carpio* is an omnivorous fish with superb taste quality and containing high quality amino acids and fatty acids [23]. The purpose of this study was to evaluate the effects of TIE supplementation on the growth and overall health of *C. carpio* fingerlings.

## 2 Materials and methods

### 2.1 Fish acclimatization and setup of trial

The present study was carried out in the laboratory at the Department of Zoology, GC University Faisalabad, Punjab, Pakistan. *C. carpio* fingerlings were acquired, from the local Fish Seed Hatchery, Faisalabad. After that, the fish were housed in 70L V-shaped tanks for 15 days to allow them to acclimatize. Fingerlings of *C. carpio* were given a salt bath (5 % NaCl) to eliminate any ectoparasites or fungus before the experiment began [24]. The fish were fed their basal feed once a day until they appeared satiated. The temperature, dissolved oxygen levels, and pH were measured daily by using the thermometer, DO metre, and pH metre (Jenway 3510). All of the fish tanks received continuous (24-h) aeration via the capillary system.

### 2.2 Extract preparation

Fresh plants of *T. indic*a were collected from Kot Sultan, a town in District Layyah of Punjab Province, Pakistan. The leaves were brought and taxonomically identified at GC University, Faisalabad. To remove dust and mud, all leaves were washed; rotten and damaged pieces were thrown away. After a few days of air drying in the shade, leaves were then completely dried in an oven at 60 °C. Following that, they were ground into a fine powder in a grinder, and refrigerated in sealed containers.

After that, mixed it with 96 % ethanol and ordinary distilled water at a ratio of 1:10 (w/v) and extracted with a mechanical shaker for 2 days [18]. A rotary evaporator was used to transform the supernatant into a paste (Labkits U-Therm International Limited, SE–CF–TDZ-WS, Hong Kong) after a 15-min centrifugation at 4000 rpm. Following which, the paste was freeze-dried, and kept in the freezer (4 °C) until needed.

### 2.3 Formulation of diets

A total of six isonitrogenous test diets were formed (Table 1, Table 2). Canola meal was used as the basal diet and TIE was added at level of 0 % (Test Diet (TD) I), 0.5 % (TD II), 1 % (TD III), 1.5 % (TD IV), 2 % (TD V) and 2.5 % (TD VI) [16,17]. Then all feed components were ground to a small size using the 0.5 mm sieve. During mixing, fish oil was progressively added. A smooth textured dough was made by adding water at a 10–15 % ratio [25]. Following which, the different TIE levels were mixed separately with the dough. Feed pellets were later produced by pelletizing the dough in a pelleting machine; the resulting pellets were then dried and kept until needed.

**Table 1:** Composition of ingredients in the test diets (%).

Ingredients	TIE^a^ (%)					
	**0**	**0.5**	**1**	**1.5**	**2**	**2.5**
Canola meal	52	52	52	52	52	52
Fish meal	15	15	15	15	15	15
Wheat flour	12	11.5	11	10.5	10	9.5
Rice polish	10	10	10	10	10	10
Fish oil	8	8	8	8	8	8
Mineral premix^b^	1	1	1	1	1	1
Vitamin premix^c^	1	1	1	1	1	1
Chromic oxide	1	1	1	1	1	1

a TIE = *Tamarindus indica* extract.

b Mineral premix kg-1: Fe: 1000 mg, Ca: 155 g, Co: 40 mg, P: 135 g, Se: 3 mg, Na: 45 g, Zn:3000 mg, Cu: 600 mg, Mg: 55 g, Mn: 2000 mg, I: 40 mg.

c Vitamin (Vit.) premix kg-1: Vit. B12: 40 mg, Vit. D3: 3,000,000 IU, Vit. A: 15,000,000 IU, Vit. C: 15,000 mg, B2: 7000 mg, Vit. K3: 8000 mg, Vit. B6: 4000 mg, Vit. Ca pantothenate: 12,000 mg, Folic acid: 1500 mg, Nicotinic acid: 60,000 mg.

**Table 2:** Proximate composition of ingredients (%).

Ingredients	Dry matter	Crude protein	Crude fat	Crude fibre	Ash	Gross Energy	Carbohydrates
**Canola meal**	90.42	37.78	3.76	6.09	9.59	3.53	42.78
**Wheat Flour**	90.89	9.95	2.98	2.47	2.08	3.12	82.52
**Fish Meal**	91.66	53.78	12.67	1.56	11.87	2.56	20.12
**Rice polish**	92.91	12.26	13.40	10.91	11.28	3.57	52.15

### 2.4 Feeding procedure and fecal collection

Twice a day, the fishes were fed with their regular diet, which accounted for 5 % of their live wet weight. After each feeding session, the tanks were drained and properly washed to remove any uneaten food particles and then refilled with fresh water. Following which, the faeces were collected via tank valves. Nutrient leaching was avoided by handling the thin faeces with care. To conduct chemical analysis, faeces were oven-dried and stored at 4 °C.

### 2.5 Growth study

Initial weights (IW) were recorded at the start of trial. The difference between IW and final weights (FW) (at end of trial) was calculated to assess the growth rate and weight gain (WG). Moreover, feed intake (FI), specific growth rate (SGR) and feed conversion ratio (FCR) were assessed by following [26].

### 2.6 Chemical evaluation of faeces, feed and fish body

Standard procedures were used to analyze the homogenized faeces, feed and body samples [27]. Feed and faeces (1 g) were dried for 12 h at 105 °C to measure their moisture content. To measure the crude protein (CP) content, a micro Kjeldahl was utilized. An electric furnace was used to measure the ash percentage. With the Soxtec (HT2 1045) device, crude fat (CF) was extracted by ether extraction technique. The total amount of energy (GE) was calculated with the help of bomb calorimeter. Crude fiber (CF) was determined by the ignition of dried lipid-free residues digested with 1.25 % NaOH and 1.25 % H_2_SO_4_. Total carbohydrates in feed were determined by the formula described below.

Totalcarbohydrates(%)=100−(CP%+CF%+Ash%+CF%+Moisture%)

### 2.7 Hematological analysis

After a trial period, fish from each tank (3 fish/tank) were tranquillized using a 150 mg/L tricane methane sulfonate to collect samples [28]. The drawn blood samples were sent to Laboratory for hematological investigation. Using commercially available 25 mm heparinized capillary tubes, packed cell volume (PCV) was calculated using a micro hematocrit centrifuge. A hemocytometer was used to calculate white blood cells (WBCs) and red blood cells (RBCs). Moreover, mean corpuscular hemoglobin (MCH), mean corpuscular hemoglobin concentration (MCHC) and mean corpuscular volume (MCV) were also determined by Ref. [26]. Hemoglobin (Hb) was determined using the method by Ref. [29].

### 2.8 Calculation of nutrient digestibility

Nutrient digestibility coefficient (ADC%) of diets were evaluated by formula as indicated by Ref. [30].

### 2.9 Statistical analysis

One-way Analysis of Variance (ANOVA) [31] to the data was done. Tukey's Honesty Significant Difference (HSD) Test was used to compare the mean differences [32]. The Co-Stat computer program (Monterey, Version 6.303, 93940 USA, PMB 320) was utilized for statistical analysis.

## 3 Results

### 3.1 Growth assessment

The general improvement of all growth parameters (WG, FCR, WG%, and SGR) was observed in *C. carpio* fed on diets supplemented with TIE (Table 3). Maximum WG (15.00 ± 0.57 g) was shown by fingerlings fed on test diet-III having 1 % TIE supplementation level. However, test diet-VI (2.5 % TIE) showed minimum WG (11.02 ± 0.21 g) as compared to control (11.71 ± 0.24 g) and other diets.

**Table 3:** Growth performance of *C. carpio* fingerlings fed on TIE supplemented canola meal.

Experimental Diets	TIE (%)	Initial Weight (g)	Final Weight (g)	Weight Gain (g)	Weight Gain (%)
Test Diet-I	0	6.64 ± 0.02^a^	18.37 ± 0.25^cd^	11.71 ± 0.24^cd^	176.47 ± 3.47^cd^
Test Diet-II	0.5	6.64 ± 0.03^a^	19.67 ± 0.13^b^	13.02 ± 0.14^b^	196.04 ± 2.71^b^
Test Diet-III	1	6.66 ± 0.04^a^	21.66 ± 0.61^a^	15.00 ± 0.57^a^	225.36 ± 7.45^a^
Test Diet-IV	1.5	6.64 ± 0.02^a^	20.91 ± 0.13^a^	14.27 ± 0.12^a^	214.96 ± 1.74^a^
Test Diet-V	2	6.51 ± 0.26a	19.00 ± 0.1^bc^	12.49 ± 0.35^bc^	192.38 ± 13.59^bc^
Test Diet-VI	2.5	6.65 ± 0.02^a^	17.67 ± 0.19^d^	11.02 ± 0.21^d^	165.59 ± 3.57^d^

At (*P<*0.05), the means of rows with different superscripts vary substantially.

The data are the averages of three replicates.

In terms of FCR, the minimum value of FCR (1.51 ± 0.01) was noted in test diet-III (1 % TIE). The TIE supplementation level of 2.5 % showed the maximum value (1.36 ± 0.05), followed by the control group (1.34 ± 0.07) (Fig. 1). The results of SGR indicated that TIE improved the SGR of fingerlings up to 2 % supplementation level than the control diet (0.45 ± 0.02 %) (Fig. 2). Maximum SGR (1.68 ± 0.03 %) was shown by fingerlings fed on 1 % TIE supplemented diet, indicating that 1 % is optimal level for TIE supplementation. While minimum SGR was noted in case of test diet-VI (2 % TIE) (1.40 ± 0.02 %).

**Fig. 1:** FCR of *C. carpio* fingerlings fed on TIE supplemented canola meal.

**Fig. 2:** SGR of *C. carpio* fingerlings fed on TIE supplemented canola meal.

### 3.2 Nutrient digestibility

The results of nutrient composition in diet of *C. carpio* when fed TIE-supplemented canola-meal revealed that the results were significantly similar (*P>*0.05) and faeces showed a substantial (*P<*0.05) variation in the nutrients (Table 4, Table 5). In terms of ADC%, 1 % TIE level gave best results for CP, CF and GE as 67.60 ± 0.83 %, 67.49 ± 0.45 % and 70.90 ± 0.56 %, respectively. The lowest results for digestibility (CP: 59.45 ± 0.34 %; CF: 59.57 ± 0.82 % and GE: 62.63 ± 0.29 %) were observed in the 2.5 % TIE level indicating maximum release of nutrients in faeces and with the least amount of nutrients being absorbed in fish body (Fig. 3).

**Table 4:** Analyzed composition (%) of (CP), (CF) and (GE) in the diet of *C. carpio* fingerlings fed on TIE supplemented canola meal.

Experimental Diets	TIE (%)	Crude Protein (%)	Crude Fat (%)	Gross Energy (%)
Test Diet-I	0	31.09 ± 0.3	9.51 ± 0.03	4.38 ± 0.02
Test Diet-II	0.5	31.08 ± 0.02	9.53 ± 0.02	4.35 ± 0.02
Test Diet-III	1	31.09 ± 0.03	9.52 ± 0.04	4.36 ± 0.03
Test Diet-IV	1.5	31.05 ± 0.05	9.48 ± 0.03	4.36 ± 0.04
Test Diet-V	2	31.05 ± 0.02	9.50 ± 0.02	4.34 ± 0.03
Test Diet-VI	2.5	31.06 ± 0.04	9.63 ± 0.24	4.34 ± 0.02

At (*P<*0.05), the means of rows with different superscripts vary substantially.

The data are the averages of three replicates.

**Table 5:** The composition (%) of (CP), (CF) and (GE) of the faeces of *C. carpio* fingerlings fed on TIE supplemented canola meal.

Experimental Diets	TIE (%)	Crude Protein (%)	Crude Fat (%)	Gross Energy (%)
Test Diet-I	0	14.73 ± 0.21^b^	4.43 ± 0.15^b^	1.90 ± 0.03^b^
Test Diet-II	0.5	13.85 ± 0.05^c^	4.04 ± 0.14^c^	1.72 ± 0.01^c^
Test Diet-III	1	12.05 ± 0.03^e^	3.7 ± 0.07^d^	1.52 ± 0.02^e^
Test Diet-IV	1.5	13.03 ± 0.8^d^	3.92 ± 0.11^cd^	1.65 ± 0.03^d^
Test Diet-V	2	14.58 ± 0.34^b^	4.39 ± 0.12^b^	1.86 ± 0.03^b^
Test Diet-VI	2.5	15.38 ± 0.20^a^	4.75 ± 0.06^a^	1.98 ± 0.03^a^

At (*P<*0.05), the means of rows with different superscripts vary substantially.

The data are the averages of three replicates.

**Fig. 3:** The apparent nutrient digestibility of *C. carpio* fingerlings fed on TIE supplemented canola meal.

### 3.3 Body composition

The body composition (CP, CF, moisture, and ash) of *C. carpio* fingerlings fed TIE supplemented in canola-meal was shown to be considerably (*P<*0.05) improved by all TIE supplementation levels when compared to the control diet, except the 2.5 % level (Table 6). However, 1 % supplementation level gave maximum protein and ash values as 63.92 ± 0.06 % and 18.60 ± 0.03 %, respectively and lowest fat (18.60 ± 0.03 %) and moisture (10.36 ± 0.04 %) contents. Minimum protein (62.20 ± 0.02 %) and ash (18.14 ± 0.02 %) contents were observed at 2.5 % level. The fat (8.47 ± 0.02 %) and moisture (11.19 ± 0.01 %) contents for 2.5 % level were highest indicating poor body composition results at this supplementation level.

**Table 6:** Whole body composition % of *C. carpio* fingerlings fed on TIE supplemented canola meal.

Experimental Diets	TIE (%)	Protein	Fat	Ash	Moisture
Test Diet-I	0	62.26 ± 0.04^d^	8.36 ± 0.03^b^	18.21 ± 0.03^e^	11.16 ± 0.02^a^
Test Diet-II	0.5	62.60 ± 0.04^c^	7.96 ± 0.01^d^	18.47 ± 0.02^c^	10.97 ± 0.03^bc^
Test Diet-III	1	63.92 ± 0.06^a^	7.12 ± 0.02^f^	18.60 ± 0.03^a^	10.36 ± 0.04^d^
Test Diet-IV	1.5	63.20 ± 0.1^b^	7.44 ± 0.03^e^	18.53 ± 0.02^b^	10.83 ± 0.14^c^
Test Diet-V	2	62.34 ± 0.04^d^	8.25 ± 0.02^c^	18.37 ± 0.01^d^	11.04 ± 0.03^ab^
Test Diet-VI	2.5	62.20 ± 0.02^d^	8.47 ± 0.02^a^	18.14 ± 0.02^f^	11.19 ± 0.01^a^

At (*P<*0.05), the means of rows with different superscripts vary substantially.

The data are the averages of three replicates.

### 3.4 Hematological indices

In general, the results of the different blood parameters (WBCs, RBCs, PCV, PLTs, Hb, MCHC, MCV and MCH) of common carp fed diets supplemented with TIE demonstrated that TIE improved the hematological indices of *C. carpio* over the control, except for the 2.5 % supplementation level (Table 7).

**Table 7:** Hematological indices of *C. carpio* fingerlings fed on TIE supplemented canola meal.

Diets	TIE (%)	RBC (10^6^mm^−3^)	WBC (10^3^mm^−3^)	PLT	Hb (g/100 ml)	PCV (%)	MCHC (%)	MCH (pg)	MCV (fl)
Test Diet-I	0	3.54 ± 0.03^e^	8.35 ± 0.04^e^	62.70 ± 0.14^e^	9.24 ± 0.02^e^	26.39 ± 0.14^e^	35.62 ± 0.14^e^	56.59 ± 0.14^e^	174.19 ± 0.78^e^
Test Diet-II	0.5	3.95 ± 0.04^c^	8.65 ± 0.03^c^	66.86 ± 0.12^c^	9.54 ± 0.03^c^	28.86 ± 0.10^c^	37.72 ± 0.23^c^	60.87 ± 0.08^c^	183.67 ± 0.28^c^
Test Diet-III	1	4.46 ± 0.02^a^	8.96 ± 0.02^a^	70.65 ± 0.13^a^	9.83 ± 0.02^a^	30.65 ± 0.03^a^	40.42 ± 0.12^a^	63.32 ± 0.60^a^	195.56 ± 0.69^a^
Test Diet-IV	1.5	4.26 ± 0.03^b^	8.83 ± 0.03^b^	69.72 ± 0.23^b^	9.74 ± 0.03^b^	30.04 ± 0.02^b^	39.80 ± 0.21^b^	62.68 ± 0.31^b^	190.28 ± 0.80^d^
Test Diet-V	2	3.75 ± 0.02^d^	8.45 ± 0.02^d^	64.50 ± 0.15^d^	9.36 ± 0.03^d^	27.25 ± 0.09^d^	36.27 ± 0.12^d^	58.60 ± 0.25^d^	177.24 ± 0.56^d^
Test Diet-VI	2.5	3.43 ± 0.02^f^	8.14 ± 0.03^f^	61.45 ± 0.19^f^	9.06 ± 0.02^f^	25.33 ± 0.18^f^	34.45 ± 0.31^f^	56.08 ± 1.20^f^	169.45 ± 0.53^f^

At (*P<*0.05), the means of rows with different superscripts vary substantially.

The data are the averages of three replicates.

Out of all test diets, test diet-III (1 % TIE) showed maximum improvement in hematological indices as WBCs (8.96 × 10^3^mm^−3^), Hb (9.83g/100 ml), RBCs (4.46 × 10^6^mm^−3^) and PCV (30.65 %). Similarly, maximum results were shown by 1 % level in case of MCHC, MCV, MCH and PLTs as 40.42 %, 195.56 fl, 63.32 pg and 70.65, respectively. Least values of blood parameters were noted in the case of test diet-VI (2.5 % TIE supplementation).

## 4 Discussion

Feed formulation techniques have been identified as the most significant productivity factors in intensive aquaculture systems [[33], [61], [66]]. Adding functional feed additives to farmed fish feed is a practical strategy to increase their health and production [5,[34], [68]]. In our study, the supplementation level of 1 % of TIE gave the best results in terms of growth performance of *C. carpio*. Similar effect was shown by purslane, as it has higher feed efficiency and palatability than other supplements; adding 0.5 % purslane to grass carp fingerlings improved their growth performance [35]. Another study investigated that dietary herbal supplements (turmeric, rosemary and thyme) that substantially enhanced the growth of Nile tilapia [36]. However, the growth parameters of gilthead seabream and Nile tilapia were negatively affected when adding more than 1 % purslane [37]. It was possible that the high levels of herbal constituents contain anti-nutritional components such as phytate and oxalate that may reduce the feed intake by the fishes. Interestingly, it was found that an inclusion level of 2.5 % TIE in our study delivered the lowest growth in common carp. In addition, variations in growth performance between fish species might be caused by factors such as species, feeding duration, and feed additive dosages [38]. Fish health is influenced by several factors, including bacterial flora, intestinal structure, and digestive enzymes activity [[39], [67]]. In addition to boosting the growth of fishes, consuming certain plants in their overall diet also improve the platibility of these fishes for human food consumption [38]. Anti-nutritional compounds found in various plants have been linked in multiple studies to poor development and digestion of feed [[40], [66]]. Although, *T. indica* was found to have no detrimental effect on feed utilization and the appetite of fishes. There was a substantial variation in weight gain and other parameters of growth between fish fed control and test diets in this study. Similar findings were reported by supplementation of *Astragalus membranaceus* on *Oreochromis niloticus* [41], *Coriandrum sativum* on *Oncorhynchus mykiss* [42]*,* and *Aloe barbadensis* on *O. mykiss* [43].

The current study found that incorporating *T. indica* to the diet improved fish growth, gut physiology, feed efficiency and digestibility of nutrients. TIE's beneficial phytochemicals (flavonoids, alkaloids, and saponin) may be responsible for the observed growth promotion and enhanced nutrient utilization in *C. carpio*. These compounds may stimulate synthesis of more digestive enzymes that enhance the development of a balanced microbiota and digestibility of nutrients. Herbs include abundant polyphenolic chemicals, which the gut flora frequently converts into readily available substances with antibacterial, anti-inflammatory and antioxidant characteristics [[67], [69]]. Nevertheless, these compounds have poor bioavailability in animals [44]. Moreover, phenolic chemicals remove the pathogenic microbes from the digestive system. Thus, the growth-promoting potential of herbal supplements may be linked to phenolic substances [[62], [64]]. Therefore, digestive enzymes stimulate the activity in the fish gut [45]. In accordance with our results, improvement in nutrient digestibility had seen in *Danio rerio* (zebrafish) [46] by dietary ginger and in *O. niloticus* by tamarind pulp extract [18].

In comparison to the fingerlings fed with the control diet (based on canola meal), the lower fat and higher protein levels were seen in fishes given the 1 % TIE supplementation level. This might be due to the fact that fishes fed with this TIE level exhibited higher protein retention (aiding in the fish's survival) and greater fat catabolism (providing energy for the fish's activity). According to Halver and Hardy [47], the fast-growing fish generally have higher retention of protein. Wafaa et al. [48] observed a drop in total body lipid with an increase in CP and ash when *O. niloticus* was fed with herbal supplements. Dietary protein significantly helps to fulfill the energy needs of fish; therefore, lipid-derived energy is utilized to conserve the proteins for growth of fish [49]. Similarly, *O. niloticus* fed with caraway seed meal or green tea displayed lower CP and ash levels and higher body fat as reported by Ref. [50]. In contrast to our results, [51] reported a significaly similar effect in carcass composition when common carps were fed with rosemary leaf powder.

Hematological parameters, including RBCs, Hematocrit, Hb concentration and WBCs are frequently used to assess fish health and antioxidative capabilities [52]. Several fish species' hematological profiles had improved after being fed with medicinal plants [53]. This research demonstrated that TIE considerably enhanced blood parameters of the common carp. Our findings are in agreement with those reported by other researches on fish fed with medicinal plant extracts, including rainbow trout [54], Nile tilapia [55], goldfish [56] and striped catfish [57]. Leukocytes are a key factor of the immune system, and their abundance can be utilized as a measure of the overall health of aquatic organisms. Interestingly, there was an increase in the total WBCs of Common carp at the end of the experimental trial. Similarly, [58] demonstrated that the common carp's total WBC count was increased with the use of immunostimulating herbal plants. It has been described that plant extracts may affect lymphoid organs, leading to increased blood cell count [59]. Moreover, according to Khieokhajonkhet et al. [60], RBCs and WBCs linearly increased (*P<*0.05) with increasing dietary turmeric extract supplementation.

## 5 Conclusion

It was demonstrated that TIE supplementation has the potential to enhance the growth, digestibility, carcass composition and hematological indices of *C. carpio*. Based on the various observations, the optimal level of TIE supplementation in the diet was 1 %. Further study is recommended to explore the detailed effects of TIE on fish health and welfare in order to enhance the sustained productivity of this species.

## Ethical statement

Ethics Review Committee of the GC university Faisalabad, Faculty of life Science approved the research design (Ref. No. GCUF/ERC/146), which was carried out in accordance with the ARRIVE principles.

## Funding

Open access funding provided by Swedish University of Agricultural Sciences.

## Data availability

Data will be available on demand.

## CRediT authorship contribution statement

**Mahnoor Saleem:** Writing – original draft. **Syed Makhdoom Hussain:** Writing – original draft, Supervision, Investigation, Formal analysis, Conceptualization. **Shafaqat Ali:** Writing – review & editing, Software, Data curation. **Muhammad Rizwan:** Writing – review & editing, Software, Data curation. **Khalid A. Al-Ghanim:** Writing – review & editing. **Jean Wan Hong Yong:** Writing – review & editing, Data curation, Funding.

## Declaration of competing interest

The authors declare that they have no known competing financial interests or personal relationships that could have appeared to influence the work reported in this paper.
